The article "Exosomes secreted from miRNA-29b-modified mesenchymal stem cells repaired spinal cord injury in rats" was published in 2019. Journal: Braz J Med Biol Res.

# Exosomes secreted from miRNA-29b-modified mesenchymal stem cells repaired spinal cord injury in rats

**DOI:** 10.1590/1414-431X20198735

**Published:** 2019-12-05

**Authors:** Tao Yu, Cunju Zhao, Shouzhi Hou, Weijie Zhou, Baoxin Wang, Yunzhen Chen

**Affiliations:** 1 Department of Spinal Surgery, Qilu Hospitial of ShanDong University, Jinan, Shandong, China; 2 Department of Orthopedics, Liaocheng People's Hospitial, Liaocheng, Shandong, China; 3 Department of Radiology, Liaocheng People's Hospitial, Liaocheng, Shandong, China

**Keywords:** miRNA-29b, Exosomes, Spinal cord injury, BMSCs

## Abstract

Exosomes, a kind of extracellular vesicle, are promising therapeutic agents for spinal cord injury (SCI). This article aimed to investigate effects of exosomes secreted from miRNA-29b-modified bone marrow mesenchymal stem cells (BMSCs) on SCI. Exosomes were extracted from BMSCs transfected with miRNA-29b or negative control (miR NC). SCI rats were injected intravenously with exosomes (control exosomes, miRNA-29b exosomes) and BMSCs (miR NC, miRNA-29b) through the tail vein. The expression of miRNA-29b in spinal cord tissues of SCI rats was detected by qRT-PCR. The hind limb motor function was evaluated by Basso Beattie Bresnahan (BBB) score. The histopathological damage and neuronal regeneration in spinal cord tissues was observed by HE staining and immunohistochemistry, respectively. The injection of miRNA-29b exosomes and miRNA-29b BMSCs both significantly increased the expression of miRNA-29b in spinal cord tissues of SCI rats (P<0.05). Compared with SCI rats, rats in the miRNA-29b exosomes and the miRNA-29b groups exhibited improved SCI, including increased BBB score, NF200 and GAP-43 positive neurons, as well as decreased contractile nerve cell numbers and GFAP positive neurons (all P<0.05). The relieving degree of SCI was significantly higher in the miRNA-29b exosomes group than in the miRNA-29b BMSCs group (P<0.05). Exosomes secreted from miRNA-29b-modified BMSCs were effective in the repair of SCI in rats.

## Introduction

Spinal cord injury (SCI) is a serious central nervous system disease that leads to severe leg dysfunction and even lifelong paralysis (1). Primary mechanical SCI can quickly trigger secondary injury and induce inflammatory response and neuronal apoptosis in the injured area (2). Subsequently, astrocyte scars and syringomyelia are formed, resulting in the inhibition of axonal regeneration and dysfunction of motor and sensory function (3). The treatment of SCI is still difficult in clinical practice due to the poor regeneration ability of neurons.

In recent years, stem cell transplantation has become a hot spot in the treatment of SCI with the development of stem cell technology. The transplantation of bone marrow mesenchymal stem cells (BMSCs) has been considered an effective therapeutic strategy for SCI, since it can inhibit inflammation and apoptosis, promote axonal regeneration and angiogenesis, reduce astrocyte scars and syringomyelia, and promote recovery of motor function (4). However, BMSCs transplantation also has some drawbacks, such as teratogenic tumorigenesis, immune rejection, pulmonary embolism, low transplantation rate, and survival rate (5,6). Exosomes (diameter: 30-100 nm) are extracellular vesicles released from cells into the extracellular space (7). As an important mediator of cell-cell interaction, exosomes can enter target cells through membrane receptors or endocytosis, and then participate in the regulation of biological information via transmitting mRNAs, non-coding small RNAs, proteins, etc. (8). Noteworthy, exosomes exert positive therapeutic effects on SCI through inhibiting neuronal apoptosis and inflammatory response (7). Huang et al. (9) found that the administration of mesenchymal stem cells (MSCs)-derived exosomes in SCI rats significantly attenuates the lesion size, as well as cellular apoptosis and inflammation in the injured spinal cord. Sun et al. (10) found that human umbilical cord MSCs-derived exosomes facilitate the healing of SCI through attenuating inflammation. Wang et al. (11) found that MSC-derived exosomes exert obvious neuroprotective effects on SCI by reducing SCI-induced A1 astrocytes and inhibiting inflammation. Therefore, exosomes are expected to be an alternative to stem cells in the treatment of SCI.

MicroRNAs (miRNAs) are a type of endogenous small RNAs with a length of 20–24 nucleotides (12). Some miRNAs contribute to the repair of damaged nerve tissues and cells, such as miR-340, miR-204, etc (13,14). BMSCs can secrete exosomes with high levels of specific miRNA by pre-transfection with specific miRNA plasmids (15). Previous studies have proven that miRNA-29 is involved in the repair of liver damage, myocardial ischemia-reperfusion injury, skeletal muscle injury, as well as human podocyte injury (16 [Bibr B17] [Bibr B18]–19). However, the regulatory role of miRNA-29 on SCI is still unclear. In this study, the effects of exosomes secreted from miRNA-29b-modified BMSCs on SCI were evaluated. Our findings may provide important clinical theoretical basis and guidance for the treatment of SCI.

## Material and Methods

### Animals

A total of 80 female Sprague-Dawley rats weighing 230–250 g were purchased from Shandong Lukang Pharmaceutical Co., Ltd. (China). Rats were routinely housed in specific pathogen-free animal rooms at 22–26°C with 40–60% humidity. All rats were given free access to water and feed. All animal experiments in this study met the requirements of the animal ethics committee of Qilu Hospitial of ShanDong University.

### Isolation and culture of BMSCs

One-month-old (100–120 g) rats were anesthetized by intraperitoneal injection of 1% pentobarbital (dose, 80 mg/kg). After being disinfected with 75% alcohol, the femur and tibia of the rat were obtained by removing the surface muscles and fascia. Bone marrow was then obtained by rinsing with Hanks solution. After 5 min of centrifugation at 170 *g* (4°C), BMSCs at the bottom of the centrifuge tube were remixed evenly with Hanks solution. Followed by 5 min of centrifugation at 1050 *g* (4°C), BMSCs were suspended in LG-DMEM cell culture medium containing 10% fetal bovine serum (FBS). Then, BMSCs were seeded in a sterile culture flask in an incubator at 37°C with 5% CO_2_. The medium was replaced with fresh medium every 2 days. After three generations, BMSCs at logarithmic growth phase were used for the following assays.

### Identification of surface markers in BMSCs

BMSCs were added into 1.5-mL centrifuge tubes at a density of 1×10^5^ cells per tube. After 5 min of centrifugation at 170 *g* (25°C), the supernatant was discarded and BMSCs at the bottom of tubes were resuspended in 100 μL D-Hanks solution. Then, FITC-labeled anti-rat CD44, PE-labeled anti-rat CD73, FIC-labeled anti-mouse IgG, and PE-labeled anti-mouse IgG antibodies were added to the tubes. D-Hanks solution was added to one of the tubes for control. All tubes were incubated at room temperature for 45 min in the dark. After washing 3 times with D-Hanks, BMSCs in each tube were analyzed by flow cytometry.

### BMSCs transfection and exosomes extraction

BMSCs were inoculated on 24-well plates at a density of 2×10^6^ cells/well. After 48 h of culturing, BMSCs were transfected with miR-29b recombinant lentiviral vector (miR-29b-LV) and recombinant LV carrying enhanced green fluorescent protein (EGFP) reporter gene (NC-EGFP-LV) (Ruibo Biotechnology Co., Ltd., China). These transfected BMSCs were named as miRNA-29b group and miR NC group, respectively. The multiplicity of infection was 20. Three days after the transfection, BMSCs were stained with DAPI for 1 h. The EGFP fluorescence was observed under a fluorescence microscope. BMSCs were collected for subsequent assays when the transfection efficiency was more than 95%. In addition, exosomes were extracted from the supernatant of each well using the Exo Quick-TC kit (SBI, USA) in strict accordance with the instructions.

### Identification of exosome protein markers by western blot

Exosomes were quantified by bicinchoninic acid (BCA) and subjected to sodium dodecyl sulfate polyacrylamide gel electrophoresis (SDS-PAGE). Then, the proteins were transferred onto a polyvinylidene fluoride (PVDF) membrane, blocked with 5% skim milk, and incubated with primary antibodies (rabbit anti-rat CD9 monoclonal antibody, ab92726; mouse anti-rat CD63 monoclonal antibody, ab108950; rabbit anti-rat CD81 monoclonal antibody, ab109201; rabbit anti-rat GAPDH polyclonal antibody, ab9485; 1:1000, Abcam, UK) for 12 h at 4°C. After washing 3 times with Tris-buffered saline and Tween 20 (TBST), the membrane was incubated with horseradish peroxidase-labeled secondary antibodies (goat anti-mouse IgG, goat anti-rabbit IgG, 1:5000, Beijing Zhongshang Jinqiao Biotechnology Co., Ltd., China) for 2 h at room temperature. After washing three times with TBST, the protein bands were detected using a Kodak film developer (Fujifilm, Japan).

### Construction of SCI model in rats

Intraperitoneal injection of 1% pentobarbital sodium at a dose of 50 mg/kg was used to anesthetize rats. Rats were placed on the operating table and disinfected. A 2-3 cm incision was made at the midline of the back using the T10 spinous process as the center. The vertebrae were exposed after the surface muscles were separated. Spinous processes and lamina were removed to fully expose the T10 spinal cord. During this procedure, the dura mater was completely preserved. Using a standard striking device, the T10 spinal cord was hit with a striking force of 2 N. The wound was stitched after being washed with penicillin saline. The successfully established rat model of SCI met the following characteristics, including congestive edema of T10 segment, twitch of tail and hind limb, and Basso Beattie Bresnahan (BBB) score less than 10.

### Grouping and intervention

A total of 100 SCI rats were randomly divided into 5 groups: SCI, control exosomes, miRNA-29b exosomes, miR NC, and miRNA-29b (n=20 per group). One hour after modeling, rats were injected intravenously with 500 μL control exosomes (secreted from miR NC BMSCs) or miRNA-29b exosomes (secreted from miRNA-29b BMSCs) at a concentration of 200 μg/mL through the tail vein. Rats injected intravenously with miR NC BMSCs and miRNA-29b BMSCs (10^7^ cells/mL, 10 μL) were enrolled as miR NC group and miRNA-29b group, respectively. Rats injected intravenously with physiological saline were enrolled as SCI group. After the injection, penicillin was injected at a dose of 2×10^5^ U/kg once a day for 3 days, and urination care was given 3 times a day until resuming active urination.

### Motor function assessment

The hind limb motor function of rats was evaluated by BBB score at 3 days, 1, 2, 4, and 8 weeks post-injection as previously described (20).

### Spinal cord tissue collection

At 3 days, 1, 2, 4, and 8 weeks post-injection, 4 rats in each group were randomly selected and deeply anesthetized. The thoracic cavity of rats was opened to expose the heart. A total of 250 mL physiological saline was perfused into the ascending aorta to adequately flush the blood in tissues. Then, 4% paraformaldehyde was perfused until the liver was whitened and stiffened. The central segment of spinal cord tissues at the injury site (T9-10, about 1 cm in length) was removed and stored in liquid nitrogen.

### Detection of miRNA-29b expression by qRT-PCR

Total RNA was extracted from spinal cord tissues 1 week post-injection using Trizol reagent according to the manufacturer's instructions. RNA samples were reversely transcribed using cDNA Reverse Transcription Kit (Applied Biosystems, USA). qRT-PCR was carried out by the Fast Start Universal SYBR Green Mastermix (Roche, USA). All primers were synthesized by Shanghai Sangon Biotech Co., Ltd., China. Primer sequences were: miRNA-29b, forward: 5′-CTGACGGAGTTCCTCCAGTTC-3′, reverse: 5′-GAGGTTCCCCGAGAAGACGAT-3′ and U6, forward: 5′-CTCGCTTCGGCAGCACA-3′, reverse: 5′-ACGCTTCACGAATTTGCGT-3′. Data were processed by the 2^-ΔΔCT^ method, and relative miRNA-29b expression was normalized to U6.

### Hematoxylin and eosin (HE) staining

Four weeks after injection, spinal cord tissues (about 0.5 cm around the injured site) were fixed with 4% paraformaldehyde for 24 h, embedded in paraffin, and sliced at a thickness of 6 μm. These tissue sections were subjected to xylene dewaxing, alcohol gradient dehydration and hydration, followed by HE staining. After being dehydrated with alcohol and xylene, sections were sealed with neutral resin and observed under an optical microscope (Olympus, Japan).

### Immunohistochemistry

Spinal cord sections were subjected to xylene dewaxing, gradient alcohol rehydration, and antigen retrieval with boiling 0.01 M citrate buffer. Endogenous peroxidase activity was eliminated by 15 min of incubation with 3% hydrogen peroxide. Then, these sections were incubated with goat serum blocking solution for 15 min at room temperature and incubated with primary antibodies (rabbit anti-rat NF200, ab8135, GFAP, ab7260, GAP-43, ab75810, 1:100, Abcam, UK) for 12 h at 4°C. After washing 3 times with PBS, sections were incubated with horseradish peroxidase-labeled goat anti-rabbit IgG (1:500, Beijing Zhongshang Jinqiao Biotechnology Co., Ltd.) for 15 min at 37°C. Followed by DAB color reaction and hematoxylin counterstaining, sections were sealed with neutral gum and observed under an optical microscope (Olympus). Positive cells were counted in 5 random fields of view.

### Statistical analysis

All experiments were repeated 3 times independently. Data were analyzed by SPSS 21.0 statistical software (USA). All quantitative data are reported as means±SD. Comparison between different groups was determined by one-way ANOVA followed by *post hoc* test (two groups). P<0.05 was considered statistically significant.

## Results

### Identification of BMSCs

After 10 days of primary culture, a large number of fusiform BMSCs were observed (Figure 1A). After three generations, the morphology of BMSCs was consistent with the morphological characteristics of BMSCs (21). Flow cytometry showed that more than 90% of BMSCs showed positive expression of CD44, CD73, and CD90 (Figure 1B). After 72 h of transfection with miRNA-29b and miR NC, more than 95% of BMSCs showed positive expression of EGFP (Figure 1C and D). Then, exosomes were extracted from transfected BMSCs. Western blot showed that miRNA-29b exosomes and control exosomes showed positive expression of CD63, CD81, and CD9 (Figure 1E).

**Figure 1:** Identification of bone marrow mesenchymal stem cells (BMSCs) and exosomes. **A**, Fusiform BMSCs were observed under a microscope after primary culture for 10 days (bar=50 μm). **B**, Positive expression of CD44, CD73, and CD90 was observed in BMSCs by flow cytometry. **C**, Enhanced green fluorescent protein (EGFP) was observed in BMSCs transfected with miR-29b-LV or NC-EGFP-LV for 72 h (bar=100 μm). **D**, Virus transfection efficiency was more than 95% in BMSCs transfected with miR-29b-LV or NC-EGFP-LV for 72 h. **E**, Positive expression of CD63, CD81, and CD9 was observed in exosomes secreted from transfected BMSCs by western blot. Data are reported as means±SD.

### miRNA-29b expression in spinal cord tissues of SCI rats

One week after injection, miRNA-29b expression in spinal cord tissues of SCI rats in each group was detected by qRT-PCR. As shown in Figure 2, the relative expression of miRNA-29b was significantly higher in the miRNA-29b exosomes group than in the control exosomes group (P<0.05). The relative expression of miRNA-29b was also significantly increased in the miRNA-29b group compared with the miR NC group (P<0.05). No significant difference for miRNA-29b expression was observed between the SCI and control exosomes and miR NC groups (Figure 2).

**Figure 2:** MiRNA-29b expression in spinal cord tissues of spinal cord injury (SCI) rats. Data are reported as means±SD. *P<0.05 *vs* SCI group; ^&^P<0.05 *vs* control exosomes; ^#^P<0.05 *vs* miR NC; ˆP<0.05 *vs* miRNA-29b exosomes (ANOVA).

### Injection of miRNA-29b exosomes accelerated the motor function of SCI rats

Reduced feeding and mobility were found in SCI rats after surgery. Severe hind-limb motor dysfunction and loss of spontaneous urinary function were also observed in SCI rats. All rats received urination care (3 times/day), and no urinary retention-induced bladder rupture occurred. The BBB scores in rats injected with BMSCs and exosomes increased with time in a time-dependent manner. The BBB scores were significantly higher in the miRNA-29b exosomes group than in the control exosomes group at 2, 4, and 8 weeks post-injection (P<0.05), and were also significantly higher in the miRNA-29b group than in the miR NC group at 1, 2, 4, and 8 weeks post-injection (P<0.05). Compared with the miRNA-29b group, the miRNA-29b exosomes group exhibited significantly higher BBB scores at 1, 2, 4, and 8 weeks post-injection (P<0.05) (Figure 3).

**Figure 3:** Basso Beattie Bresnahan (BBB) scores of rats at 3 days, 1, 2, 4, and 8 weeks post-injection. Data are reported as means±SD. *P<0.05 *vs* SCI group; ^&^P<0.05 *vs* control exosomes; ^#^P<0.05 *vs* miR NC; ˆP<0.05 *vs* miRNA-29b exosomes (ANOVA).

### Injection of miRNA-29b exosomes alleviated histopathological damage in spinal cord tissues of SCI rats

Severe structural disorder, rupture of the vessel wall, and neuronal edema were observed in spinal cord tissues of SCI rats. The boundary between the white matter and the gray matter was blurred, and enhanced neuronal nuclear staining was also observed in the spinal cord gray matter. At 4 weeks post-injection, the number of contractile nerve cells in the SCI group was significantly decreased by the injection of BMSCs or exosomes (P<0.05). In addition, the number of contractile nerve cells in the miRNA-29b exosomes group was significantly lower than in the control exosomes group (P<0.05). When compared with the miR NC group, a significantly lower number of contractile nerve cells was found in the miRNA-29b group (P<0.05). Noteworthy, the miRNA-29b exosomes group exhibited a significantly lower number of contractile nerve cells than the miRNA-29b group (P<0.05) (Figure 4).

**Figure 4:** Contractile nerve cells were observed in spinal cord tissues of spinal cord injury (SCI) rats by HE staining at 4 weeks post-injection (×400, bar=100 μm). Arrows indicate contractile nerve cells. Data are reported as means±SD. *P<0.05 *vs* SCI group; ^&^P<0.05 *vs* control exosomes; ^#^P<0.05 *vs* miR NC; ˆP<0.05 *vs* miRNA-29b exosomes (ANOVA).

### Injection of miRNA-29b exosomes promoted neuronal regeneration

Neurofilament protein 200 (NF200), growth-associated protein-43 (GAP-43), and glial fibrillary acidic protein (GFAP) are three important proteins involved in neuronal regeneration. Immunohistochemical staining showed that relative low expression of NF200 and GAP-43 was observed in spinal cord tissues of SCI rats. The injection of BMSCs or exosomes significantly increased the expression of NF200 and GAP-43 in SCI rats at 2, 4, and 8 weeks post-injection (P<0.05). In addition, the expression of NF200, GAP-43, and GFAP was significantly higher in the miRNA-29b exosomes group than in the control exosomes group (P<0.05), and also significantly higher in the miRNA-29b group than in the miR NC group at 1, 2, 4, and 8 weeks post-injection (P<0.05). Compared with the miRNA-29b group, the miRNA-29b exosomes group exhibited significantly higher NF200 and GAP-43 expression (P<0.05) (Figure 5A and B). In contrast, the expression changes of GFAP in spinal cord tissues of SCI rats in the 5 groups were just the opposite to NF200 at 1, 2, 4, and 8 weeks post-injection (P<0.05) (Figure 5C).

**Figure 5:** NF200 (**A**), GAP-43 (**B**), and GFAP (**C**) positive cells (brown) were observed in spinal cord tissues of spinal cord injury (SCI) rats by immunohistochemistry at 3 days, 1, 2, 4, and 8 weeks post-injection (×500, bar=100 μm). Data are reported as means±SD. *P<0.05 *vs* SCI group; ^&^P<0.05 *vs* control exosomes; ^#^P<0.05 *vs* miR NC; ˆP<0.05 *vs* miRNA-29b exosomes (ANOVA).

## Discussion

The pathophysiological changes of SCI mainly include two stages: primary injury and secondary injury (22). Primary injury involves spinal cord hemorrhage, nerve cell membrane rupture, as well as blood-brain barrier disruption caused by external traction or compression (23). Secondary injury is a series of chain reactions after primary injury, which involves local blood flow disorder, tissue ischemia and hypoxia, inflammatory cell infiltration, and nerve cell necrosis. Secondary injury results in further enlargement of the spinal cord injury area, more nerve cell death, and even nerve fiber deformation (24). In general, secondary injury is more severe and more difficult to manage than primary injury.

At present, many animal experiments and clinical studies have confirmed that BMSCs transplantation achieves a certain therapeutic effect on SCI (25,26). Most studies believe that BMSCs play an important role on the repair of SCI by secreting various regulatory factors (26,27). However, the clinical application of BMSCs transplantation is very limited due to low survival rate and differentiation rate *in vivo* (28). In 2010, Lai et al. (29) demonstrated for the first time that neurotrophic factors and nerve growth factors are exosomes secreted by MSCs. Exosomes are extracellular vesicles that contain a variety of biologically active substances, such as proteins, mRNAs, and miRNAs. Exosomes are able to promote intercellular communication through exchanging protein and genetic information (30). Teng et al. (31) confirmed that exosomes secreted by MSCs promote neovascularization, and inhibit inflammation in myocardial ischemic injury. Huang et al. (9) reported that exosomes secreted by MSCs promote functional recovery of SCI by relieving apoptosis and the inflammatory response, and stimulating angiogenesis. These findings indicate that the intervention of exosomes secreted by MSCs is a potential therapeutic strategy for SCI. In this research, results were consistent with the above previous studies, and further illustrate that the injection of exosomes was effective in the treatment of SCI.

miRNAs are a class of small non-coding RNAs, which exert important regulatory effects on cell biological behavior (32). Our results indicated that the injection of miRNA-29b exosomes was able to accelerate the repair of SCI. In recent years, accumulated studies have shown that exosomes carrying miRNAs exert key repairing effects on damaged tissues. For example, Shen et al. (12) indicated that the brain injury in intracerebral hemorrhage rats is attenuated by the transplantation of exosomes carrying miR-133b. The mechanism involved in this process is that miR-133b can activate ERK1/2/CREB pathway, thereby inhibiting neuronal apoptosis and neurodegeneration. Chen et al. (15) showed that exosomes derived from miR-223 inhibitors-transfected BMSCs protect liver damage by regulating NLRP3 and caspase-1. Our findings were consistent with previous studies, and illustrated that the injection of miRNA-29b exosomes relieved the SCI in rats. Furthermore, we also found that the injection of miRNA-29b exosomes significantly increased NF200 and GAP-43 positive neurons, and decreased GFAP positive neurons. NF200 is a skeletal structure of neural cells and axons (33 [Bibr B34]). GAP-43 is a specific phosphoprotein on vertebrate nerve cell membrane that is considered a marker for synaptic plasticity, neuronal development, and regeneration (34). GFAP, a cytoskeletal protein, is the major component of glial cells (35). In the early stage of SCI, GFAP expression is up-regulated, and some cytokines are secreted to promote axonal regeneration. However, in the late stage of SCI, a large number of hyperplastic glial scars may inhibit the growth of axons (36). Since these three proteins can reflect the degree of neuronal regeneration in spinal cord tissues of SCI rats, our results further indicated that miRNA-29b exosomes can relieve SCI by regulating the expression of NF200, GAP-43, and GFAP.

In conclusion, the injection of exosomes secreted by miRNA-29b-modified BMSCs repaired SCI in rats. The relevant mechanism might be associated with the regulation of proteins involved in neuronal regeneration, such as NF200, GAP-43, and GFAP. Exosomes secreted by miRNA-29b-modified BMSCs may be a promising therapeutic agent for SCI in clinical practice.
